# Construction of a Physical and Medical Care Integrated Model for the Elderly in the Community Based on Artificial Intelligence and Machine Learning

**DOI:** 10.1155/2022/3678577

**Published:** 2022-02-25

**Authors:** Zongyou Yang, Siyong Xia, Sheng Feng

**Affiliations:** ^1^Department of Physical Education, Chongqing Jiaotong University, Nanan, 400074 Chongqing, China; ^2^School of Physical Education, Southwest University, Beibei, 400700 Chongqing, China; ^3^Physical Education Department of Chongqing Medical and Pharmaceutical College, 401331 Chongqing, China

## Abstract

With the increasingly serious population aging, economic system transformation, and social transformation, the elderly have an increasingly strong demand for the elderly care service industry, but the development of China's elderly care service industry started late, and there are still many problems. For how to build a better elderly care service model, under the current situation of shortage of elderly care resources, community elderly care may become a solution. By analyzing the status quo, existing problems and development trends of home-based care services in Hangzhou's community, and learning from foreign experience, it explores the establishment of a “integrated physical, medical, and nursing care” community health management model for the elderly and provides a perfect solution for the development of Hangzhou's community elderly care services countermeasures and suggestions for mode operation. Based on the evaluation, problem analysis, and empirical research on the current situation of home care services in Hangzhou communities, this paper draws on relatively mature community care practices, proposes to build a community elderly health management model that combines medical care and care, and improves and innovates the overall design and medical care of the elderly service model measures for the health management of the elderly in the integrated community. The experimental results of this study show that, according to the demand for elderly care services, elderly people in need of care account for 86.6%, 79.5%, and 68.4% of the elderly population, especially in the areas of medical care, life care, and housekeeping services.

## 1. Introduction

### 1.1. Background

During the “Twelfth Five-Year Plan” period, Hangzhou's population aging has intensified, and the elderly population has increased by 340,200. As of the end of 2015, the city's elderly population was 1.5 million, accounting for 20.86% of the registered population, showing the “four modernizations” trend of aging, aging, empty nesting, and disability. On the one hand, with the elderly, the elderly with disabilities, dementias, and chronic diseases have increased. Single elderly care services or medical services have been unable to meet the elderly's health and elderly needs. The comprehensive needs of the elderly for basic living care, disease prevention, and rehabilitation care are increasing day by day. There is an urgent need to establish a multilevel system. At present, the intelligent home-based elderly care model under development may provide a comprehensive service system. It does provide elderly care at home and provide supporting facilities and services inside or around the community: the service system and the provision of diversified service content to meet the growing, escalating, and personalized healthcare needs of the elderly. On the other hand, the miniaturization, empty nesting, and weakening of family care functions have made the elderly not getting the care they deserve. However, the ideal state of the elderly for the elderly is health and security, care for their lives, and spiritual exchanges. Therefore, society, communities, and institutions are required to provide service support for the elderly.

### 1.2. Significance

At present, the problem of population aging in our country is becoming more and more prominent, but the traditional home-based care model in China can no longer meet the needs of the elderly for the elderly, and our country's elderly care industry is still in its infancy, with small business scale and low degree of industrialization structure, single industrial structure and few product types, and poor service quality and low benefit of pension industry; the government policy environment is not ideal. And all aspects are actively exploring new types of elderly care models suitable for China's national conditions, to meet the needs of the elderly in our country. Through analysis and field investigation of the current status and existing problems of the elderly care facilities in our country, at the same time, we will study and learn from the latest successful case experience of foreign elderly care real estate. Starting from the spiritual and cultural needs of the elderly that are easily overlooked by the public, we will explore a way that can satisfy all of them. In terms of needs, the old-age care model that can meet the national conditions of our country is expected to provide some reference and reference for practitioners in the planning, architectural design, investment, and operation of future retirement communities. At the same time, it can also provide reference for relevant decision-making, operation, and management departments and enrich the content of the construction of elderly care facilities, which is of great significance for solving the increasingly serious elderly care problems in our country.

### 1.3. Related Work

With the continuous development of society and the continuous renewal of information technology, there are more new formats for the elderly care service industry.

Ahn et al.'s research uses grounded theory and content analysis to conduct in-depth, semistructured interviews with 10 nationally recognized experts on the use of lean management in healthcare organizations. The purpose is to understand if and how lean management can be used to achieve breakthrough improvements in performance. The results of his experiments reveal some differences in how experts define breakthrough improvement and illustrate the value of human-centered design thinking, alone or as a complement to lean management, in achieving breakthrough improvements in healthcare organizations. However, there is a lot of redundant data in his research [1]. Bethea A is based on preexisting conditions and declining physiological reserves in older adults that often complicate healthcare delivery in this population; the design model enables the NP to initiate admissions and coordinate hypoacuity patients under the supervision of a trauma attending physician daily care. His study sought to compare outcomes in older patients whose care was coordinated by trauma NP (TNP) versus nontraumatic NP (NTNP) services. These clinical and economic results have proven helpful in substantiating the care provided by TNP at research facilities. However, his experiments lack a certain amount of objective factual basis [2]. Chen et al., based on social support theory and differential order pattern, explored the underlying mechanism and boundary conditions of the relationship between social interaction and life satisfaction among the rural elderly. On the one hand, it explores the mediating role of psychological well-being in the relationship between social interaction and life satisfaction, and on the other hand it examines whether emotional support moderates the effects of social communication on mental health. Using structural equation modeling, they analyzed data from 658 rural older adults in China and concluded that the relationship between social communication and mental health was negatively moderated by emotional support. Finally, the implications for management theory and practice are discussed. However, they did not propose specific countermeasures [3].

### 1.4. Innovation

The innovation of this article is as follows. (1) In meeting the basic needs of medical care and healthcare for the elderly, it combines the retirement community with educational facilities, such as colleges and kindergartens, to enrich the spiritual and cultural needs of the elderly, so as to meet the needs of the elderly and all aspects of the needs to improve the quality of life for the elderly. (2) Following the forefront of the development of the elderly care industry, using technical methods such as satisfaction description, factor analysis, and regression model, based on the analysis of the status quo of community home (CH) care services, evaluation analysis, and supply and demand forecasting, innovatively cut from the perspective of the integration of medical care and care, we proposed a CH care service model that combines medical care and care.

This paper is structured as follows: the introduction part of this article introduces the trend of population aging and then leads to the importance of community elderly health management model construction; the method part introduces the related algorithms of artificial intelligence and machine learning, including XGBoost algorithm, decision tree algorithm, and logistic regression model. The experimental part designs the overall design of the community's elderly health management model, constructs service evaluation indicators, and builds an elderly care service model with the medical care structure; the analysis part analyzes the community's demand for elderly care services and the macroevaluation and draws a conclusion: community elderly health. The construction of a management model is very meaningful.

## 2. Artificial Intelligence and Machine Learning Related Algorithms

### 2.1. XGBoost Algorithm

XGBoost has strong abstract data analysis and processing capabilities, and its efficient, flexible, and accurate prediction capabilities make it the most popular algorithm in the field of machine learning [4]. It is also widely used in fields including statistical learning, data analysis, artificial intelligence, etc. The loss function of XGBoost is shown in the following equation:

(1) $$\begin{array}{c} \text{L}\left(\emptyset \right)=\sum_{\text{i}=1}^{\text{n}}\text{l}\left(\hat{{\text{y}}_{\text{i}}},{\text{y}}_{\text{i}}\right)+\sum_{\text{k}=1}^{\text{k}}\rho \left({\text{f}}_{\text{k}}\right). \end{array}$$

The predicted value $\hat{y_{i}}$ of the model is shown in formula (2).

(2) $$\begin{array}{c} \hat{y_{i}}=\emptyset \left(x_{i}\right)\\ =\sum_{k=1}^{K}f_{k}\left(x_{i}\right). \end{array}$$

Because XGBoost is an additive model, that is, given an input *x*_*i*_, the output is to add the predicted values of *k* regression trees, so the model predicts the score; it is the cumulative sum of the $\hat{y_{i}}$ scores of each tree.

*ρ* is a regularization term, which defines the function of model complexity; see (3) for details. It adds the complexity of all *k* trees to the objective function to prevent the model from overfitting.

(3) $$\begin{array}{c} \rho \left(f\right)=\gamma T+\frac{1}{2}\delta \sum_{j=1}^{T}\omega_{j}^{2}. \end{array}$$

The complexity of defining a tree is usually composed of two parts: the number of leaf nodes *T* and the weight of leaf nodes *ω*_*j*_, *γ*, and *δ* are the penalty coefficients set manually, so for the regularization term, the previous part is the decision. For the complexity of the tree structure, the latter part is the complexity of the predicted value of the decision tree [5].

(4) $$\begin{array}{c} {\hat{y_{i}}}^{\left(t\right)}\sum_{k=1}^{t}f_{k}\left(x_{i}\right)={\hat{y_{i}}}^{\left(t-1\right)}+f_{t}\left(x_{i}\right). \end{array}$$

As shown in formula (4), the prediction result of sample *i* after the *t*-th iteration is the sum of the prediction results of the previous *t* − 1 trees and the *t*-th regression tree.

XGBoost algorithm is mainly used for the preference of different elderly groups for health management services in the construction of community elderly health management model. It can be divided according to gender and age stage and score the preference and satisfaction.

### 2.2. Decision Tree Algorithm

The difficulty of decision tree construction is how to segment features. The purpose is to use a fixed measurement standard to calculate multiple features for classification after decision branching. For the application of decision tree feature segmentation, the commonly used methods include information gain, information gain ratio, Gini coefficient, and mean square deviation. Assuming that the proportion of the m-th sample in the current sample set *D* is *p*_*m*_ (*m* = 1, 2,…, *y*), the information entropy of *D* is defined as

(5) $$\begin{array}{c} \text{Ent}\left(\text{D}\right)=-\sum_{\text{m}=1}^{\left|\text{y}\right|}p_{m}log_{2}p_{m}. \end{array}$$

The smaller the value of Ent(*D*), the higher the purity of *D*. Assuming that the discrete attribute *a* has *X* possible values {*a*_1_, *a*_2_,…, *a*_*X*_}, if the sample set is divided by *a*, *X* branch nodes will be generated [6]. According to the above formula, the information entropy of *D*^*X*^ can be calculated, so the “information gain” obtained by dividing the sample set *D* by attribute *a* can be calculated:

(6) $$\begin{array}{c} \text{Gain}\left(D,a\right)=\text{Ent}\left(D\right)-\sum_{X=1}^{X}\frac{\left|D^{X0}\right|}{\left|D\right|}\left(\text{Ent }D^{X}\right). \end{array}$$

Generally speaking, the greater the information gain, the higher the purity. *a*_*∗*_ = argmax Gain(*D*, *a*) is used for attribute division. Since information gain has a preference for attributes with more values, in order to reduce this adverse effect, the concept of gain rate is proposed to classify the optimal attributes:

(7) $$\begin{array}{c} {\text{Gain}}_{\text{ratio}\left(D,a\right)}=\frac{\text{Gain}\left(D,a\right)}{\text{IV}\left(a\right)}. \end{array}$$

Among them

(8) $$\begin{array}{c} \text{IV}\left(a\right)=-\sum_{X=1}^{X}\frac{\left|D^{X}\right|}{\left|D\right|}\log_{2}\frac{\left|D^{X}\right|}{\left|D\right|}. \end{array}$$

CART (Classification and Regression Tree) uses the Gini index to classify attributes, and the purity of data set *D* can be measured by the Gini value:

(9) $$\begin{array}{c} \text{Gini}\left(D\right)=\overset{\left|y\right|}{\underset{m=1}{\sum }}\underset{m^{\prime }\neq m}{\sum }p_{m}p_{m}^{\prime }\\ =1-\overset{\left|y\right|}{\underset{m=1}{\sum }}p_{m}^{2}. \end{array}$$

In general, the Gini index reflects the probability that two random sample categories in the data set are inconsistent: the smaller the value, the higher the purity. The higher the purity, the better the classification and processing effect of the data set. The best feature is usually selected with the smallest Gini index, which can make the community health management model provide differentiated and accurate services for different groups. The Gini index of attribute *a* is

(10) $$\begin{array}{c} \text{Gini}\_\text{index}\left(D,a\right)=-\sum_{X=1}^{X}\frac{\left|D^{X}\right|}{\left|D\right|}\text{Gini}\left(D^{X}\right). \end{array}$$

The traditional decision tree model has a preference for attributes with more numerical values and can only handle discretely distributed features, and there is no pruning process. At the same time, the entropy model is used, which contains a large number of logarithmic operations, and the time cost is high.

### 2.3. Logistic Regression Model

Logistic Regression is an easy-to-implement and excellent performance classification model for linear separable problems, and it is one of the most widely used models [7]. It limits the decision function to a certain condition and is generally used to solve the binary classification problem. In this study, it can be used to estimate the possibility that different groups in the community need health and elderly care services. The logistic regression algorithm is an extension of the traditional linear model.

First construct a traditional linear regression model:

(11) $$\begin{array}{c} \mu =b+w_{1}x_{1}+\cdots +w_{p}x_{p}=w^{T}x+b. \end{array}$$

In this model, the value range is (−∞, +∞).

Logistic regression is a machine learning method used to solve the problem of binary classification (0 or 1), which is used to estimate the possibility of something, such as the possibility of a user buying a commodity, the possibility of a patient suffering from a disease, and the possibility of an advertisement being clicked by the user.

Suppose the two categories of the binary classification problem are *y* = 1 and *y* = 0, and the probability of *y* = 1 is *π*, that is, *π* = *p*(*y* = 1). In the logistic regression model, the difference between *π* and *η* is sigmoid function relationship, namely,

(12) $$\begin{array}{c} \pi =\frac{1}{1+{\text{e}}^{-\mu }}\;\mu \in \left(-\infty ,+\infty \right). \end{array}$$

Through the sigmoid function, (−∞, +∞) can be projected onto (0, 1) to indicate the probability of whether the event will occur, so as to complete the binary classification problem. The binary classification problem of logistic regression can finally be expressed as

(13) $$\begin{array}{c} \left\{\begin{array}{c} 0\;\pi <0.5,\\ 1\;\pi >0.5. \end{array}\right) \end{array}$$

The training process of the logistic regression binary classification model is the process of finding (*w*, *b*) through an appropriate method.

(14) $$\begin{array}{c} P\left(y=1\right)=\frac{1}{\;1+e^{-\mu }}\;\\ =\frac{1}{1+e^{-\left(w^{T}x+b\right)}}\;\\ =\frac{e^{-\left(w^{T}x+b\right)}}{1+e^{-\left(w^{T}x+b\right)}}\\ =\;\pi ,\\ p\left(y=0\right)=1-p\left(y=1\right)\\ =\frac{1}{1+e^{-\left(w^{T}x+b\right)}}\\ =1-\pi . \end{array}$$

For ease of presentation, suppose *θ*=(*w*, *b*). The maximum likelihood estimation method is commonly used to solve (*w*, *b*). Given the data set {(*x*_*i*_, *y*_*i*_)}_*i*=1_^*m*^, the likelihood function expression is

(15) $$\begin{array}{c} L\left(\theta \right)=\overset{m}{\underset{i=1}{\prod }}{\left(\pi \right)}^{y_{i}}{\left(1-\pi \right)}^{1-y_{i}}. \end{array}$$

Defining the loss function *J*(*θ*) of logistic regression as the opposite of the logarithm of the above formula, we can get

(16) $$\begin{array}{c} \text{J}\left(\theta \right)=-\text{lnL}\left(\theta \right)\\ =-\overset{m}{\underset{i=1}{\sum }}\left(y_{i}\text{ln}\left(\pi \right)+\left(1-y_{i}\right)\text{ln}\left(1-\pi \right)\right). \end{array}$$

Therefore, maximizing the likelihood function is equivalent to minimizing the loss function. In the usual research, the value of *θ*=(*w*, *b*) is often obtained by minimizing the loss function *J*(*θ*).

## 3. The Overall Design of the Health Management Model for the Elderly in the Community

On the basis of the previous analysis, this chapter designs a set of Hangzhou CH care service model based on the domestic and foreign service practice experience, aiming to construct a scientific and feasible service model that realizes the integration of “medicine” and “nourishment” [8].  Figure 1 shows the CH-based care service structure of the combination of medical and elderly care.

### 3.1. Construction of Evaluation Indicators for CH Care Services

#### 3.1.1. Design Goals of Evaluation Indicators

Carry out an overall evaluation of Hangzhou CH care service and understand its overall level of supply and demand and its shortcomings, so as to promote its development and improvement.

#### 3.1.2. Design Principles of Evaluation Indicators

*(1) Multilevel Evaluation*. One is to conduct an overall evaluation of Hangzhou CH care services at the macrolevel, and the second is to analyze the problems of the current system from the microlevel. At the macrolevel, the evaluation parameters include positive indicators and negative indicators. The positive indicators include the professional level of service organization, whether the service functions are complete, and whether the service team and fund are in place, and the negative indicators include the imperfection of market mechanism and the lack of government leadership. At the microlevel, the evaluation parameter is mainly the satisfaction with healthcare services.

*(2) Quantitative and Qualitative Evaluation*. Adopt a combination of qualitative and quantitative evaluation methods to give full play to the advantages of the two and complement each other. Quantitative evaluation is to use mathematical methods to collect and process data and make value judgment of quantitative results for the evaluation object. Qualitative evaluation is to directly make value judgment of qualitative conclusion for the evaluation object according to the evaluator's observation and analysis of the evaluation object's usual performance, reality, and state.

#### 3.1.3. The Specific Content of the Evaluation Index

*(1) Macroindicators*. The establishment of a macro index evaluation system is to evaluate the overall level of home care services in Hangzhou communities. The core content of macro indicators includes service organizations, functions, teams, funds, government, markets, social organizations, etc. The macrolevel institutional pension resource allocation evaluation index system is shown in Table 1.

*(2) Microindicators*. At the microlevel, the micro index system is established by adding the concept of satisfaction, and the current model is evaluated by measuring whether the supply of home care services and facilities in the community meets the demand. Through interviews and questionnaire surveys of the elderly in the community, the satisfaction data of this part is obtained, and a microlevel satisfaction index system is established according to the needs and content of the elderly's concentrated attention and in accordance with the principles of science and control [9]. The satisfaction option uses a Likert five-point scale, using 1, 2, 3, 4, and 5 to represent very dissatisfied, less dissatisfied, fair, more satisfied, and very satisfied. At the same time, all survey content reflects the average. It is subjective satisfaction.  Table 2 shows the evaluation indicators of microlevel institutional resource allocation.

### 3.2. The Construction of a CH-Based Elderly Care Service Model Combining Medical and Elderly Care

The “Combination of Medical Care” model takes into account both medical and maintenance aspects of elderly care. Compared with traditional elderly care methods, medical elements are placed in a more important position, and this model not only covers daily care, spiritual comfort, and style. Entertainment services, etc., cover medical and healthcare services such as medical rehabilitation, healthcare, diagnosis and treatment of illness, and hospice care. In addition, the medical services in this medical care integration model are all services with a certain professional level, which need to meet the professional level of hospitals above the first level, and they must have complete facilities and medical items and have a certain amount of space guarantee and hardware [10]. The guarantee of facilities such as medical service equipment requires a professional medical team in software. In the construction of the medical care integration model, it is necessary to systematically introduce the related system policies, main body composition, and service resources. Based on the operating experience of old-age care methods in western developed countries, this study expounds the CH-based care service model combining medical care and care from the perspectives of individuals, communities, and systems. Its main structure is shown in Figure 2.

#### 3.2.1. Personal Level

From an individual perspective, there are mainly six types of elderly who need medical care, namely, those with chronic diseases, those with relapse-prone diseases, the elderly who are frail, and those who have just recovered, and those who are terminally ill. Moreover, according to the health status of the elderly, elderly people who cannot take care of themselves need to go to institutions for the elderly and receive medical services, while those who are in good health, those who have basic health, or those who are unhealthy but able to take care of themselves are provided with integrated medical care services in the community more convenient. In terms of service content, the combination of medical care and elderly care for the elderly who choose the CH care model is very extensive, including home daily life services, (psychological) physical therapy healthcare services, spiritual comfort psychological counseling services, cultural entertainment, and social activities, etc. By embedding in the community platform, the function improves the efficiency of resource allocation and promotes the development of elderly care services.

#### 3.2.2. Community Level

Community services are continuous and universal, which is very necessary for the development of elderly care services. For an elderly person, he will have a variety of elderly care services and care needs. If only relying on elderly care institutions and families to provide elderly care services, it is far from reaching the requirements, and it is not in line with the current level of social and economic development in our country to adapt. In addition, as the main daily activity area for the elderly, the community plays an important role in the care of the elderly and is an important channel to realize various elderly care measures [11]. At the community level, it will have broad prospects to build a medical care integrated service system and establish a community-based elderly care service model that integrates medical and elderly care. With the community as the supporting platform, it is possible to build a comprehensive model that realizes the integration of medical and nursing care, that is, to build a platform around the community, coordinate various resources and various forces, and develop the active participation of the government, society, institutions, and individuals in policy design. On the basis of diversified collaboration and personal self-management, it is built into a step-by-step service process with fixed coverage. The CH care service model based on the combination of medical and elderly care is shown in Figure 3.

At the macrolevel, the community is a comprehensive support body, which can make full use of the functions and roles of the community, construct a multidimensional comprehensive service model, develop a community elderly care service management system, and use the Internet to achieve service links. At the microlevel, communities are integrated into various regions and multisource resources. We should make full use of existing resources, absorb government and social resources, and coordinate to build a community-based service model that integrates medical care and nursing care.

#### 3.2.3. Institutional Level

Currently, the supply of CH care services mainly comes from government departments, enterprises, and institutions, as well as social organizations and residents' organizations. The model of multiagent collaboration requires that each entity be in a scientific system, form a competitive or cooperative relationship, and finally reach a coordination mechanism. The institutional design of the CH-based care model that combines medical care and care also requires multiparty cooperation. Both internal and external cooperation must be strengthened and overall management should be carried out.

The construction of the institutional level of the CH care service model combining medical care and elderly care needs to fully study the diversified needs of the elderly, establish demand orientation, continuously strengthen the division of labor, establish a formal and informal service system framework, and finally build it into a diversified system community-based home care service system that integrates with networked medical care. In addition, the establishment of such a system includes not only a formal care system based on community services and various services provided by various service stations, but also an informal care system based on elderly families [12]. These two care systems must achieve coordination, cooperation, and mutual complementation and jointly form a comprehensive CH care service system that combines medical care and care. The home care service system in Hangzhou urban communities is shown in Figure 4.

In the context of population aging and aging development, the demand for CH care services is increasing year by year. Under such circumstances, the state has introduced relevant policies and increased the supply of people, finances, and materials, making the community's home care services have a lot of room for improvement. In order to further study the overall level and operating conditions of home care services in Hangzhou communities, the problems and bottlenecks were found. This chapter aims to scientifically evaluate Hangzhou CH care services by building a multilevel evaluation index system, combining qualitative and quantitative ones.

## 4. Construction of the “Integration of Physical, Medical, and Nursing Care” Community Health Management Model for the Elderly

### 4.1. Service Demand Analysis of CH-Based Care

#### 4.1.1. Overall Assessment of CH-Based Care Needs

The survey shows that elderly people of different age levels, marital status, income, education, and physical health have different needs for CH care services. Therefore, in the specific process of developing services, it is necessary to treat the elderly and fully understand and master the diversified needs and develop targeted services for the elderly on this basis. In general, Hangzhou is currently increasing its support for CH care services, and the various services of CH care also largely meet the needs of most elderly people [13]. The government's financial expenditures for elderly care services are also continuously increasing, and pension funds are constantly being enriched, and the demand for elderly care is also growing rigidly and diversified, which puts forward higher requirements for elderly care services. The growth of the elderly population in Hangzhou from 1961 to 2020 is shown in Figure 5.

According to the research summary, it can be seen that the current CH care services in Hangzhou are mainly developed around the following needs of the elderly, namely, life care, housekeeping services, medical care, spiritual comfort, counseling services, and cultural and sports entertainment. The priority analysis of the needs of the elderly for home care services is shown in Table 3.

As can be seen from the above table, the order of the elderly's needs for CH care services is cultural and sports entertainment, medical care, spiritual comfort, housekeeping services, life care, and consulting services. The elderly have a higher demand for culture, sports, and entertainment, accounting for 68.9%. This requires communities to fully develop and utilize various cultural and sports facilities, establish activity teams and bases, and provide conditions and places for the elderly to carry out cultural, sports, and entertainment activities [14]. Next, medical care is also relatively high in demand. Because the elderly often suffer from various chronic diseases and physical defects, their elderly physical health needs the guidance and care of a team of medical professionals. Consulting services are ranked last among these six needs. However, in the current society, the elderly will also face family disputes and rights disputes. Providing consulting services and legal assistance for the elderly is also an important measure of CH care services and can meet the special needs of this part of the elderly to a large extent. Therefore, in the policy formulation and top-level design of CH care services, the government can fully consider the actual needs of the elderly and establish and improve relevant and targeted institutional mechanisms based on the needs. The descriptive analysis of the demand intensity of home care services is shown in Table 4.

In the survey of the service demand intensity, it can be found that the demand intensity of housekeeping services, medical care, and problem entertainment is relatively concentrated, all around 2.5, reflecting the relatively general demand for these services by the elderly. The intensity of the need for spiritual comfort is 3.41, which shows that the elderly have higher and higher requirements for spiritual life, and this requirement not only is met by recreational and sports, but also requires more professional psychological counseling and service teams. The help of the elderly is to diagnose and serve some of the psychological conditions faced and produced by the elderly. At the same time, the demand for life care and counseling services is the lowest, both less than 2. This is because some elderly people can take care of themselves and do not need special living care. On the other hand, the elderly have some problems and are not always accustomed to them. Yu consults and seeks help from the outside world.

#### 4.1.2. Analysis of the Characteristics of CH Care Needs

In the survey samples, the chi-square test was performed on factors such as gender, age, education level, home ownership, marital status, economic status, living style, health status, and social security status. The interactive analysis is shown in the following table. The data shows that the individual increase of elderly objects and their willingness to accept home care services have a significant impact. The interaction analysis between the individual characteristics of the survey subjects and their willingness to accept home care services is shown in Figure 6.

*(1) Home Care Needs of Elderly People of Different Genders*. The results of the survey show that the average life expectancy of older women is higher, and the proportion of widows will also increase. However, their educational level and income status in the elderly are lower than those of men. At the same time, due to illness or weakened functions, the elderly female population has a relatively high demand for medical services. However, given the constraints of their economic level, their medical needs cannot be completely solved with the help of market forces. In addition, counseling services and spiritual comfort services for female elderly groups are also at a relatively high level of demand, which to a certain extent is related to the social status and economic conditions of female elderly groups, because in society, these female elderly groups are in high demand. The disadvantaged position has a relatively high demand for rights protection. At the same time, the elderly female groups have relatively high psychological sensitivity, and they also have greater reflections on the relationship between family members and physical illnesses, which are likely to cause mood swings. Therefore, the elderly female groups have a greater need for spiritual comfort. The percentage (%) of elderly women's needs for specific service items for home care is shown in Table 5.

In contrast, the elderly male population has a greater demand for medical care, and there is a higher level of demand for both life care and housekeeping services. The reason for this is that the basic life skills of elderly men are less mastered than women. After the death of their spouse, the living care of elderly men often becomes a big problem, and it is difficult to find suitable people to help solve. Therefore, in terms of the demand for CH care services, there is also more demand for basic living care.

*(2) According to the Self-Care Ability, Home Care Needs*. According to the self-care situation of the elderly, the elderly who need care include those who cannot take care of themselves at all or part of their lives. The elderly who do not need care are those who have the ability to take care of themselves [15]. According to the demand for elderly care services, elderly people in need of care have relatively high demand for CH care services in all aspects, especially in the areas of medical care, life care, and housekeeping services. The demand accounts for 86.6%, 79.5%, and 68.4%.  Table 6 shows the percentage (%) of the demand for home care services for the elderly who cannot fully take care of themselves.

Elderly people with different self-care abilities and different health conditions have different content and demand levels for elderly care services. Under the current background of increasing aging, the elderly who cannot take care of themselves at all need to be given more care and consideration. The government should make targeted measures in policy design and strengthen the guarantee of funds, equipment, and human resources and do a good job in the supply of reference materials services. At the same time, it can also be seen from the demand percentage results that, at present, the needs of the elderly for community health management are not completely consistent, and the situation is more complex. Especially at the moment of the shortage of elderly care service resources and professionals, it is necessary to take new technologies as the guarantee, such as intelligent technologies represented by artificial intelligence and machine learning, to build an adaptive, flexible community health management mode that accurately meets the needs.

### 4.2. Macrolevel Evaluation of CH Care Services

#### 4.2.1. Service Institutions of CH-Based Care Services

As of 2019, Hangzhou has built 234 service points in the communities of various districts and counties, employing 32,000 people and serving 219,000 elderly people, accounting for 6.9% of the city's elderly. There are about 90,000 elderly people who purchase services at their own expense, accounting for about 41.1%. There are 283 home care centers for the elderly, where about 8,000 elderly people enjoy home care services, there are 339 catering service points for the elderly, and 34,000 elderly people receive services. In the years from 2014 to 2019, day care service organizations have grown from 83 to 283, and service employees have grown from 2,108 to more than 8,000. The total investment in the construction of new beds in Hangzhou from 2014 to 2019 is shown in Table 7.

### 4.3. Microlevel Evaluation of CH Care Services

The microlevel evaluation is mainly based on the survey and analysis of samples and conducts a survey and quantitative analysis of the satisfaction of the elderly with CH care services.

#### 4.3.1. Sample Description Analysis

The survey adopted random sampling to survey the elderly in 17 communities in 5 districts and counties of Hangzhou. A total of 520 questionnaires were sent out and 500 valid questionnaires were returned. The survey results are shown in Table 8.

#### 4.3.2. Descriptive Analysis of Satisfaction

The survey results of senior citizens' satisfaction with CH care services are shown in Figure 7.

The survey shows that the elderly are highly satisfied with the timeliness of social work services, social work attitudes, the convenience of community living facilities, the convenience of community shopping, and the convenience of going to the hospital for medical treatment. This is related to the current development status of the community. The sex is greater. At the same time, the elderly have expressed more dissatisfaction with the timeliness of social work services, community psychological counseling, and community medical care. This also reflects the shortcomings of the current CH care services and the lack of “medicine” and “nurturing” fully integrated defects. In addition, while 25.5% are very satisfied with CH care services, there are also 6.8% very dissatisfied, which also reflects the current imbalance in the quality and service quality of the community's home care service staff.

## 5. Conclusions

At present, there are problems such as imbalance between supply and demand for home care services in Hangzhou community, imperfect combination of medical care and elderly care, and unreasonable use of resources, which can no longer meet the current needs of healthy elderly care and long-term care development. Based on the research, analysis, and evaluation of the current status of CH care services in Hangzhou, this research carried out a research on the medical care integration model based on the practical experience of foreign CH care services and proposed a CH care service that combines medical care and care. The construction of the service model is envisaged, and the feasibility argument has been carried out. It has filled a certain gap in the research in the field of integrating medical and nursing elements into CH care services.

## Figures and Tables

**Figure 1:** CH care service structure combining medical care and elderly care.

**Figure 2:** System display diagram of the home-based elderly care model in the combined medical and elderly communities.

**Figure 3:** CH care service model based on the combination of medical and elderly care.

**Figure 4:** Hangzhou urban CH care service system.

**Figure 5:** Growth of the elderly population in Hangzhou from 1961 to 2020.

**Figure 6:** Interaction analysis between the individual characteristics of the survey respondents and their willingness to accept home care services.

**Figure 7:** Satisfaction of CH-based care services.

**Table 1:** Macrolevel institutional pension resource allocation evaluation index system.

Aspect	Core indicators	Specific indicators	Evaluation method
Positive index	Service organization	(1) Community service agencies for the elderly	Quantitative evaluation
		(2) Home care center	
		(3) Elderly meal service points	
	Service function	(1) Life care services	Quantitative evaluation
		(2) Basic medical and healthcare services	
		(3) Places for cultural and sports activities	
	Service team and funds	(1) CH care workers	Quantitative evaluation
		(2) Service subsidies	

Negative index	Lack of government dominance	(1) Narrowing service connotation	Qualitative evaluation
		(2) The government's responsibilities are diluted	
	The market mechanism is not sound	(1) The profit margin of the enterprise is small	Qualitative evaluation
		(2) Insufficient vitality of private capital	
		(3) Unbalanced supply and demand	

**Table 2:** Evaluation indicators of microlevel institutional resource allocation.

Microevaluation	Specific indicators
Satisfaction of CH care services	Completeness of medical facilities
	Adequacy of medical staff
	Medical level
	Timeliness of caregiver services
	Attitudes of caregivers
	Professionalism of caregiver service

**Table 3:** Priority analysis of the needs of the elderly for home care services (multiple choices).

Project	Sample	Frequency	Percentage%	Sorting
Life care	238	112	47.1	5
Housekeeping	238	129	54.2	4
Medical care	238	157	66.0	2
Spiritual comfort	238	146	61.3	3
Consultation service	238	92	38.7	6
Sports and entertainment	238	164	68.9	1

**Table 4:** Descriptive analysis of demand intensity of home care services.

The level of demand for life care	Minimum	Max	Mean	Standard deviation
Degree of demand for housekeeping services	238	112	47.1	5
Degree of demand for medical care	238	129	54.2	4
The degree of need for spiritual comfort	238	157	66.0	2
Degree of demand for consulting services	238	146	61.3	3
The degree of demand for culture, sports, and entertainment	238	92	38.7	6
The level of demand for life care	238	164	68.9	1

**Table 5:** Percentage of elderly women's demand for specific service items for home care services (%).

	Medical care	Life care	Housekeeping	Sports and entertainment	Consultation service	Spiritual comfort
It is necessary now	80.8	50.6	43.9	56.3	62.3	65.7
It will be necessary later	12.3	21.1	27.0	21.5	24.9	19.3
No need	6.9	28.3	29.1	22.2	12.8	15.0

**Table 6:** Percentage of demand for home-based care services for elderly people who cannot fully take care of themselves (%).

	Medical care	Life care	Housekeeping	Sports and entertainment	Consultation service	Spiritual comfort
It is necessary now	86.6	79.5	68.4	53.7	52.4	60.7
It will be necessary later	6.5	14.1	22.6	14.4	22.7	29.3
No need	6.9	6.4	9.0	31.9	24.9	10.0

**Table 7:** The total investment in the construction of new beds in Hangzhou from 2014 to 2019.

Years	Number of newly added beds	New beds in social elderly care institutions	Municipal financial and welfare subsidies (10,000)	District, county, and neighborhood government investment (10,000)	Social investment (ten thousand)	Total
2014	10206	1670	5, 000	8,496	37,552	51048
2015	10050	6973	5, 000	14,427	31,929	51356
2016	10769	7976	5, 000	18,700	28,781	52481
2017	9305	6229	5,000	54,622	28,584	88206
2018	7982	4980	5,000	98,834	23,767	127601
2019	4055	3672	3, 372	24,547	16,259	44178

**Table 8:** Basic situation of survey samples.

Variable		Value	
Gender	Male	180	36
	Female	320	64

Age	60–69 years old	32	6.5
	70–79 years old	94	18.8
	80–89 years old	265	53
	Over 90 years old	109	21.7

Spouse situation	No	20	4
	Divorce	3	0.5
	Passed away	415	83
	Alive	62	12.5

Physical conditions	Take care of yourself	261	52.2
	Partially unable to take care of himself	191	38.3
	Totally unable to take care of himself	48	9.5

How to live before moving into a nursing home	Live with children	132	26.5
	Live with wife	135	27
	Live alone	228	45.5
	Other	5	1

## Data Availability

No data were used to support this study.
